# Potential of Landsat 8 OLI for mapping and monitoring of soil salinity in an arid region: A case study in Dushak, Turkmenistan

**DOI:** 10.1371/journal.pone.0259695

**Published:** 2021-11-15

**Authors:** Elif Günal, Xiukang Wang, Orhan Mete Kılıc, Mesut Budak, Sami Al Obaid, Mohammad Javed Ansari, Marian Brestic

**Affiliations:** 1 Department of Soil Science and Plant Nutrition, Faculty of Agriculture, Tokat Gaziosmanpasa University, Tokat, Turkey; 2 College of Life Science, Yan’an University, Yan’an, China; 3 Geography Department, Arts and Science Faculty, Tokat Gaziosmanpasa University, Tokat, Turkey; 4 Soil Science and Plant Nutrition Department, Agricultural Faculty, Siirt University, Siirt, Turkey; 5 Department of Botany and Microbiology, College of Science, King Saud University, Riyadh, Saudi Arabia; 6 Department of Botany, Hindu College Moradabad, Mahatma Jyotiba Phule Rohilkhand University, Bareilly, India; 7 Department of Plant Physiology, Slovak University of Agriculture, Nitra, Slovakia; Harran Üniversitesi: Harran Universitesi, TURKEY

## Abstract

Soil salinity is the most common land degradation agent that impairs soil functions, ecosystem services and negatively affects agricultural production in arid and semi-arid regions of the world. Therefore, reliable methods are needed to estimate spatial distribution of soil salinity for the management, remediation, monitoring and utilization of saline soils. This study investigated the potential of Landsat 8 OLI satellite data and vegetation, soil salinity and moisture indices in estimating surface salinity of 1014.6 ha agricultural land located in Dushak, Turkmenistan. Linear regression model was developed between land measurements and remotely sensed indicators. A systematic regular grid-sampling method was used to collect 50 soil samples from 0–20 cm depth. Sixteen indices were extracted from Landsat-8 OLI satellite images. Simple and multivariate regression models were developed between the measured electrical conductivity values and the remotely sensed indicators. The highest correlation between remote sensing indicators and soil EC values in determining soil salinity was calculated in SAVI index (r = 0.54). The reliability indicated by R2 value (0.29) of regression model developed with the SAVI index was low. Therefore, new model was developed by selecting the indicators that can be included in the multiple regression model from the remote sensing indicators. A significant (r = 0.74) correlation was obtained between the multivariate regression model and soil EC values, and salinity was successfully mapped at a moderate level (R2: 0.55). The classification of the salinity map showed that 21.71% of the field was non-saline, 29.78% slightly saline, 31.40% moderately saline, 15.25% strongly saline and 1.44% very strongly. The results revealed that multivariate regression models with the help of Landsat 8 OLI satellite images and indices obtained from the images can be used for modeling and mapping soil salinity of small-scale lands.

## Introduction

Land degradation is one of the most important global concern of the 21^st^ century, negatively affecting the productivity of agricultural lands, sustainability of ecosystem services and food security as well as the quality of life. Soil salinity is one of the most important land degradation process, which threats agricultural productivity and sustainability in arid and semi-arid regions [1–3]. In addition, soil salinity causes dispersion of soil aggregates and thus negatively affects engineering properties of soils and air and water movements [2]. Natural processes and human activities are responsible for soil salinity. The accumulation of soluble salts in groundwater on soil surface causes primary soil salinity in arid and semi-arid regions where precipitation is less than evaporation, while irrigation of lands with high mineral content and drainage problems causes secondary soil salinity [4]. The lands exposed to primary and secondary salinity worldwide are 955 and 77 Mha, respectively [5]. Salinization problem continue to occur/affect 2×10^6^ ha land every year [6]. Therefore, reclamation of salt-affected lands is important to meet the food and fiber demands of increasing world population and ensure sustainable and economic use of agricultural lands. Hence, mapping and monitoring of soil salinity are necessary to define the nature of salt-affected soils and to generate accurate and reliable information about the spatial and temporal expansion of salinity.

Mapping and monitoring of spatial and temporal changes in soil salinity using remote sensing methods can be faster, cheaper and more effective than traditional methods [7, 8]. Therefore, the relationship between salt concentration and spectral properties of salt-affected soils has been focused in remote sensing studies for decades [4, 9]. The presence of salts on soil surface is determined by remote sensing data or directly by efflorescence and salt crusts, or indirectly by identification of plant species and their growth patterns. The lack of vegetation or irregular vegetation pattern help in the identification of salt-affected areas [4]. However halophytes may constrain the identification of salt-affected areas and complicate the use of remote sensing techniques in monitoring soil salinity [10].

The data sources used in remote sensing consist of aerial photographs, multispectral and hyperspectral sensors that records data in visible and infrared spectral ranges [11, 12]. Multispectral satellite sensors have been extensively studied over the past 20 years due to their ability to map and monitor surface salinity at various spatial and temporal scales [13–15]. Soil salinity in Konya province of Turkey was estimated and mapped successfully (R^2^ = 0.95) using an empirical model constructed by reflectance values of Landsat 5 images and field sampling [16]. Similarly, Shrestha [17] successfully modeled the relationship between spectral reflection values and EC measurements of soils in the north east of Thailand using Landsat ETM+ bands and multiple regression analysis. Bannari et al. [18] applied quadratic polynomial regression between visible, near-infrared (VNIR) and short-wave infrared (SWIR) spectral bands of Sentinel MSI images and in situ measurements in an arid region of Bahrain. Higher model prediction coefficient value was obtained in distinguishing soil salinity using SWIR band compared to the other bands. In addition, various researchers precisely distinguished salt separation by using numerical indices obtained by converting different spectral bands of multispectral images into a single band [19, 20].

Soil salinity negatively affects vegetation; however, traditional salinity assessment methods used in remote sensing often ignore vegetation information [10]. Remotely sensed data in sparsely distributed vegetation cover includes vegetation and soil response [21], which may cause confusion in interpretation of the data. Therefore, reflectance from vegetation has been used as an indirect indicator to improve the prediction accuracy of soil salinity using a variety of vegetation indices such as soil-adjusted vegetation index (SAVI) [22], normalized differential salinity index (NDSI) [23], vegetation soil salinity index (VSI) [24], and modified soil adjusted vegetation index-salinity index (MSAVI-SI) [25]. Similar to the vegetation indices, spectral soil salinity indices have also been developed to detect and map soil salinity [23, 26–28].

Potential relationships between soil properties and remotely sensed data can be determined with simple linear regression models [1]. However, the impact of environmental factors such as soil moisture, surface roughness, soil organic matter content, and salt mineral type etc. on soil salinity reduces the success of linear regression approaches in remote sensing studies [29]. The multivariate linear regression (MLR) uses multiple independent variables instead of simple linear methods. Therefore, MLR provides more valid and powerful explanatory models in determining soil salinity [4, 30]. Dushak is one of the important agricultural production regions for Turkmenistan, which faces the soil salinity problems in agricultural production areas. Therefore, cheaper, and faster mapping and monitoring of soil salinity is required to increase the agricultural production, determine better land management practices, prevent and reduce land degradation. The use of remote sensing data and linear regression models increase the prediction of soil salinity in a shorter time and with less cost. In line with these goals, the main purpose of this study was to map the spatial distribution of soil salinity for an agricultural farm by developing linear regression equations between spectral salinity, vegetation and moisture indices developed using the Landsat 8 bands and images. The models obtained in this study will enable the prediction and mapping of soil salinity in similar lands in the region.

## Materials and methods

### Study area

The study area consists of 1014.58 ha land located between 60.096–60.136 east longitudes and 37.136–37.103 north latitudes in the Southeast of Dushak town of Ahal Province in Turkmenistan. The average elevation above sea level of the area is 245 m. Agricultural production in Turkmenistan is mostly carried out in the Tejen region, where the study area is located. Higher annual evaporation compared to the precipitation, and the saline character of groundwater in the region [31] caused an increase in salt content of soils in the area.

The climate is distinctly continental and arid (a desert climate), and the study area receives little rainfall throughout the year. Annual average total precipitation is 189 mm, and according to Köppen and Geiger, the climate is classified as BWk. The least amount of precipitation occurred in July (0 mm), while long term average highest precipitation occurred in March with an average of 41 mm (Table 1). The months with no or the lowest precipitation are the months with the highest temperatures. The average annual temperature is 15.7° C. The hottest month of the year is July with an average of 29.0°C, while January has the lowest average temperature of the year (2.2°C). The average annual evaporation from water surface varies from 2000 to 2300 mm [32].

**Table 1:** Average long-term climate data of the Dushak city, Turkmenistan.

Attributes/Months	1	2	3	4	5	6	7	8	9	10	11	12
**Mean Temperature (°C)**	2.2	4	8.9	15.3	21.6	26.2	29	27.1	22.7	16.7	9.8	5.1
**Min. Temperature (°C)**	-3.3	-1.4	2.9	8.6	14.3	18.2	21.1	18.8	14.2	8.8	3	0
**Max. Temperature (°C)**	7.7	9.4	14.9	22.1	29	34.2	36.9	35.5	31.2	24.6	16.7	10.2
**Precipitation (mm)**	25	22	41	33	20	3	0	0	2	9	15	19

### Methods

The methodology used in the study consisted of five stages, i.e., 1) collecting soil samples from the field and laboratory analysis, 2) obtaining satellite image for the preparation of remote sensing data sets and calculating reflection values and vegetation and salinity index values, 3) calculation of correlations between measured soil EC values and remote sensing dataset, 4) testing of linear regression models, and 5) mapping the most successful model and examining the spatial distribution of soil salinity.

### Soil sampling and laboratory analysis

Fifty soil samples were collected at approximately corners of fifty 330 × 330 m grid pattern from 0–30 cm soil depth on January 15, 2019 (Fig 1). The location of each sampling point was recorded using a global positioning system. Soil samples were analyzed for electrical conductivity (EC). Soil samples were dried at room temperature and then passed through a 2 mm sieve before laboratory analysis. The EC values of soil samples were measured in the saturation pastes [33]. The point database of the measured soil EC values and coordinates of sampling points was created in the geographic information systems software ArcGIS 10.5. [34]. Resolution of Landsat images is 30 m; therefore, the digital map of the field measurements was created with the same resolution using ordinary kriging (Eq 1) method. This procedure allowed to compare the data sets with the same resolution. The EC values of sampling points were retrieved from the created map and used as the dependent variable in the statistical analyses.

**Fig 1:** Landsat 8 OLI reflectance spectra curves of different soil electrical conductivity values in the study area.


$$ϒ\;(h)=\frac{1}{2N(h)}\sum_{i=1}^{N(h)}\left[Z(x_{i})-Z{\left(x_{i}+h\right)}^{2}\right].$$ Eq 1

where Z(xi), ϒ(h), and N(h) are measured soil properties at the location of xi, the variogram for a lag distance h between Z(xi) and Z(xi + h), and the number of data pairs, respectively.

### Remote sensing data and processing

Landsat 8 OLI satellite image was used in the study. The date of Landsat 8 OLI Level 1T image used in the study was January 31, 2019 (Path/Row: 159/34, UTM WGS1984 Zone: 41). The Landsat 8 image was radiometrically calibrated and converted to surface reflectance using the SAGA GIS [35]. General characteristics of the Landsat 8 OLI image downloaded were given in Table 2. Panchromatic, Cirrus and Thermal infrared bands were not used in the study. The buildings in the farmland were masked and excluded from the evaluation. The study area boundary map was subset with OLI image using the shape file, and the image was made ready for analysis in ERDAS-Imagine® (version 2014) software [36].

**Table 2:** Specifications of spectral bands of Landsat-8 OLI [37].

Satellite Platform	Landsat 8
Sensor	OLI
Image Extent	180 × 185
Spatial Resolution utilized bands	30 m
Repeat Cycle	16 days
Utilized Bands	Band 2 (Blue: 0.45–0.51 μm)
	Band 3 (Green: 0.53–0.59 μm)
	Band 4 (Red: 0.64–0.67 μm)
	Band 5 (NIR: 0.85–0.88 μm)
	Band 6 (SWIR 1: 1.57–1.65 μm)
	Band 7 (SWIR 2: 2.11–2.19 μm)

Some salinity and vegetation indices suggested in the literature were calculated to determine and map the soil salinity following the necessary pre-processing of satellite images. The equations of the indices are given in Table 3. Spectral bands of OLI image and indices calculated from the bands were opened in grid format in geographic information systems (GIS) and overlapped with the coordinates of soil EC sampling points. The reflection values of the salinity and vegetation indices calculated with the bands of satellite image using the point database were extracted in the GIS software, and the remote sensing data set for OLI was processed for statistical analysis.

**Table 3:** Equations used to analyze spectral soil salinity and vegetation indices.

Salinity indices	Band Ratios	Reference
Normalized difference salinity index	$NDSI=\frac{\left(R-NIR\right)}{\left(R+NIR\right)}$	[23]
Vegetation soil Salinity index	VSSI = 2 x G– 5 x (R +NIR)	[24]
Brightness index	$\mathrm{BI}=\sqrt{R^{2}+{NIR}^{2}}$	[23]
Salinity index-1	$SI=\sqrt{\left(BxR\right)}$	[23]
Salinity index-2	$SI=\sqrt{\left(GxR\right)}$	[23]
Salinity index-3	$\mathrm{SI}=\sqrt{{(G}^{2}+R^{2}+{NIR}^{2}})$	[26]
Salinity index-4	$\mathrm{SI}=\sqrt{{(G}^{2}+R^{2}})$	[26]
Salinity index-5	$SI=\frac{B}{R}$	[13]
Salinity index-6	$SI=\frac{\left(B-R\right)}{\left(B+R\right)}$	[13]
Salinity index-7	$SI=\frac{\left(GxR\right)}{B}$	[13]
Salinity index-8	$SI=\frac{\left(BxR\right)}{G}$	[27]
Salinity index-9	$SI=\frac{\left(NIRxR\right)}{G}$	[27]
Moisture stress index	$MSI=\frac{\left({SWIR}_{1}\right)}{NIR}$	[38]
Normalized Difference Vegetation Index	$NDVI=\frac{\left(NIR-R\right)}{\left(NIR+R\right)}$	[23]
Normalized Difference Water Index	$NDWI=\frac{\left(NIR-SWIR1\right)}{\left(NIR+SWIR1\right)}$	[39]
Soil Adjusted Vegetation Index (L = 0.5)	SAVI = (1 + L) × NIR −	[24]
	R/L + NIR + R	

B: Blue; G: Green; R: Red; NIR: Near Infrared.

### Statistical analysis

One of the important assumptions in linear statistical analysis is normal distribution of the data. Therefore, the distribution of the data was checked with the Kolmogorov-Smirnov test. Normality test results revealed that the distribution was not normal; therefore, the data were approximated to the normal distribution by logarithmic transformation (Table 4).

**Table 4:** The results of Kolmogorov-Smirnov test.

	Statistic	df	Sig.	Transformed variable	Statistic	df	Sig.
EC	0.228	50	0.000	logEC	0.11	50	0.173

The relationships between soil EC values and remote sensing data set were analyzed with Pearson correlation test. Thus, the ability of OLI images to determine soil salinity was compared. The highest significant correlation in the correlation test was modeled by linear and multiple linear regression analysis. In regression modelling, soil EC values were defined as dependent, and band and spectral index reflection values were defined as independent variables. The validity of linear model was tested with analysis of variance and coefficient of determination (R^2^) and using residual scatter plot with ANOVA analysis. The R and R^2^ values close to 1.0 indicate a strong relationship and a model that shows a good fit [40]. In addition, higher values of the regression sum of squares values compared to the residuals sum of squares values in the variance analysis indicates the success of the models.

## Results

### Data analysis

The EC value ranges from 3.0 dS m^-1^ (slightly saline) to 35.6 dS m^-1^ (very strongly saline), and mean EC value was 11 dS m^-1^ which corresponded to strong soil salinity [33]. The coefficient of variation (65.17%) indicated that the salinity of soils in the study area is highly variable (Table 5).

**Table 5:** Descriptive statistics of electrical conductivity (EC) values [41].

	Unit	Min.	Max.	Mean	Std. Error	Coefficient of variation (%)
Soil EC (0–30 cm)	dS m^-1^	3.00	35.4	11.0	7.14	65.17

The correlations between the logEC values of the soil samples and the bands of Landsat 8 OLI sensor and the reflections of the indices derived from these bands were given in Table 6. The correlations between logEC values and NIR wavelength and BI, SI3, SI9 and VSSI indices were not significant, while logEC values had statistically significant correlation with all other variables (Table 6). The correlation between logEC and SAVI (-0.54), NDVI (-0.51), SI6 (-0.47), SI5 (-0.46), and VSSI (-0.16) was negative while the correlation with remaining variables was positive. The highest correlation between the bands of OLI sensor was obtained in the Red band (0.48), and the correlation of others was close to the Red band. The Blue and SWIR2 bands had a very close correlation (0.47). The lowest correlation was obtained in the NIR band. The highest positive and negative correlations between logEC values and indices calculated from OLI sensor data were recorded with SAVI (-0.54) NDSI (0.52), and NDWI (-0.51) indices, which were considered moderately successful in determining the soil salinity.

**Table 6:** The correlations between wavelengths and indexes calculated from OLI sensor and logEC values.

Remote Sensing Data	Blue	Green	Red	NIR	SWIR1	SWIR2					
	0.47**	0.44**	0.48**	-0.27	0.40**	0.47**					
Soil Indices	NDSI	BI	SI1	SI2	SI3	SI4	SI5	SI6	SI7	SI8	SI9
	0.52**	0.08	0.36*	0.47**	0.19	0.47**	-0.46**	-0.47**	0.47**	0.48**	0.16
Vegetation Indices	NDVI	VSSI	SAVI								
	-0.51**	-0.16	-0.54**								
Moisture Indices	NDWI	MSI									
	-0.44**	0.45**									

**Correlation is significant at the 0.01 level

* Correlation is significant at the 0.05 level.

### Investigation of spectral characteristics of Landsat images

Spectral reflections for EC values of soil samples taken from areas covered with different surface cover densities have been shown in Fig 1. The increase in salt content of soils caused an increase in the amount of spectral reflection. The increase in the amount of reflection in satellite images with the increase of soil salinity is parallel with the findings reported by Bouaziz et al. [28]. The data indicated that high reflectance characteristic of highly saline soils is important in modeling and mapping soil salinity with remote sensing data sets. Similar to our findings, distinctive absorption behaviors have been reported at visible (Blue, Green, Red) and near infrared (NIR) spectral ranges in the spectral signatures of saline soils [42]. Significant correlation was also reported between this characteristic spectral behavior and salt content of soils; thus, spectral signature of saline soils has been used in the quantitative determination of saline soils using remote sensing [14].

The lowest reflection values were recorded at visible wavelengths (VIS), while the highest reflection value was obtained in the SWIR1 band at infrared wavelengths. The reflection in SWIR2 wavelength was sharply decreased in sensor. The findings of Hu et al. [14] who reported similar spectral curves for saline soils are in accordance with our results. In addition, no obvious regularity was recorded between the reflection in the SWIR2 band and the salt content of soils with different EC readings (Fig 1). The highest reflection in sensor for high salt content was recorded in the SWIR1 band. Similarly, Bannari et al. [18] who used data of Sentinel MSI sensor, reported that the reflection in SWIR1 band is higher compared to visible and NIR bands, therefore, can be used successfully in determining and mapping soil salinity. The reflection in visible wavelengths was small, while the amount of reflection increased in the infrared wavelengths. Bouaziz et al. [28] and Fourati et al. [43] were also reported similar increase and decreases in reflections.

#### Model development and performance assessment

The strongest correlation (-0.54) among the entire remote sensing data set was calculated in the SAVI vegetation index produced using the Landsat 8 OLI image. Therefore, this index is used as an independent variable for simple linear regression. The model summary indicated that correlation coefficient (r) between the observed and predicted values of dependent variable and determination coefficient (R^2^) in the dependent variable were explained by the regression model (Table 7). Soil salinity can be estimated successfully (p <0.001) (Table 8) with the model created, while model can explain about 29% (R^2^:0.29) of the total variation in salinity. Higher value for sum of residuals squares than the sum of regression squares indicates that the explanatory power of model is not sufficient. Multiple variables were included in the modeling to increase the explanatory power of the regression models. A summary of the multiple regression models is given in Table 7. In model 2, variables with correlation coefficients above 50% were included in the modeling. This model was able to explain 28% of the total variance in soil EC. In the third model, the independent variables with p<0.05 were included in the modeling and the others were excluded. Accordingly, 11 independent variables with p<0.05 were included in the modeling. Model 3 was able to explain 55% (R^2^ = 0.55, p<0.000) of the total variance in the dependent variable. In the ANOVA test, higher values for regression sum of squares than the sum of residual squares indicates that the model can successfully predict. In addition, normal distribution for the scatter plot of the residuals indicates that the model is reliable (Fig 2).

**Fig 2:** Scatter plot of the regression residuals.

**Table 7:** Summary of linear regressions model.

Model	Variable	Regression	Std. Error of the Estimate	*p-Value*
		Coefficient		
1	Intercept	1.582	0.221	<0.001***
	SAVI	-3.465		<0.001***
		**R = 0.54 R**^**2**^ = 0.29**		
2	Intercept	1.516	0.2247	0.004**
	SAVI	-2.303		<0.001***
	NDVI	-0.066		<0.05*
	NDSI	0.307		0.003**
		**R = 0.53 R**^**2**^ = 0.28**		
3	Intercept	11.532	0.1956	0.007**
	BLUE	-95.731		0.009**
	SWIR1	-10.384		0.008**
	SWIR2	-22.364		0.005**
	SI5	-23.588		0.009**
	SI6	73.388		0.005**
	SI7	32.809		0.007**
	SI8	45.363		0.002**
	SI9	12.539		0.005**
	BI	12.018		0.001**
	MSI	15.760		0.001**
	SAVI	0.138		0.009**
		**R = 0.74 R**^**2**^ = 0.55**		

**Table 8:** The results of ANOVA test for linear regression.

Model		Sum of Squares	df	Mean Square	F	Sig.
1	Regression	0.863	1	0.863	17.611	0.000
	Residual	2.353	48	0.049		
	Total	3.216	49			
2	Regression	0.892	3	0.297	5.887	0.002
	Residual	2.324	46	0.051		
	Total	3.216	49			
3	Regression	1.757	11	0.160	4.160	0.000
	Residual	1.459	38	0.138		
	Total	3.216	49			

#### Spatial distribution of soil salinity

The most successful result in linear regression models was calculated with model 3 and soil salinity of the land was mapped using model 3. Spatial distribution of EC produced by the linear model developed using the model 3 was shown in Fig 3. The salinity map indicates that soil EC values varies between 0.65 and 39.56 ds m^-1^ in the study area. The coverage of different salt level classes in the study area was given in Table 9. Non saline soils cover 220.22 ha (21.71%), slightly saline soils cover 302.18 ha (29.78), moderately saline soils cover 318.55 ha (31.40), strongly saline soils cover154.73 ha (15.25%) and very strongly saline soils cover 14.57 ha (1.44%) land. Very strongly saline areas are mostly located in the northeastern part of the study area (Fig 3). Spatial distribution maps show that the salinity is higher than 4 ds m^-1^ in 48.51% of the study area. Salinity is higher especially in the northern and eastern parts of the study area. The salinity in south, southwest, and west sections is lower than 4 ds m^-1^ and constitutes 51.49% of the area.

**Fig 3:** Spatial distribution of EC values in the study area. The data to generate the figure was obtained from Landsat (http://landsat.visibleearth.nasa.gov/).

**Table 9:** Coverage area of different electrical conductivity (EC) classes in the study area estimated from the model maps.

EC Class	Area ha	Area %
0–2 Non saline	220.22	21.71
2–4 Slightly saline	302.18	29.78
4–8 Moderately saline	318.45	31.40
8–16 Strongly saline	154.73	15.25
>16 Very strongly saline	14.67	1.44
Masked Area	4.32	0.43
Total	1014.58	100

## Discussion

The success of linear regression methods in modeling soil EC with remote sensing methods was investigated. In the first step, the highest correlation between the remote sensing dataset and soil EC values was modeled for univariate regression analysis. SAVI index had the highest correlation (r = -0.54); thus, it was used in the modeling. The surface salt content of soils in agricultural lands was successfully determined (P<0.001) using the linear regression method with the SAVI index produced from OLI sensors. In contrast to our findings, Fourati et al. [43] recorded poor correlation between SAVI index and Landsat 8 images in determining saline areas of southeastern Tunisia. The findings obtained in this study are consistent with those reported by Alhammadi & Glenn [44] and Allbed et al. [45]. Therefore, the SAVI is considered as a promising vegetation index in determining the salt content of surface soils in both bare and vegetation-covered agricultural lands where soil salinity is a problem. However, the SAVI index explains only 29% of the total variance, which reduces the success of the model. Therefore, more variables were added to the model to increase the explanatory power of new model. Model 3 was created with eleven variables and was able to successfully explain 55% of the total variance in the study area at 99% significance level. In this study, a stronger model was developed compared to the models reported by Shrestha [17] and Shamsi et al. [9]. In addition, the results indicated that the success of linear regression model, which is obtained by adding more variables, is higher compared to the univariate regression models. Bouaziz et al. [28] and Noroozi et al. [46] also improved the success of the models with a similar procedure. The inclusion of different salt and vegetation indices to the model increased the potential of model explaining soil salinity. Similarly, Allbed et al. [45] and Guo et al. [10] emphasized that the inclusion of salt indices and vegetation indices in the model increases the success of single satellite image bands to determine salt-affected soils by remote sensing.

The information on spatial distribution of salinity is important to determine better management decisions with the goal of maximizing agricultural productivity in saline soils [41]. This study revealed that soil salinity could be successfully predicted with medium resolution satellite images and multivariate regression models. Thus, soil salinity in the study area will be monitored in the future and will be able to provide helpful data for decision-support systems to the land use planners in effective planning. In addition, remote sensing technology is very advantageous in terms of saving cost, labor, and time in development of best management plans.

## Conclusion

This study showed that linear regression model produced by the combination of Landsat 8 OLI bands and spectral indices developed quickly and successfully determines the soil salinity of a saline agricultural land in Turkmenistan. Univariate linear regression analysis explained 29% of the total variation in the study area, while multivariate regression analysis explained 55% of the spatial variation in soil salinity of the study area. The salinity classification of the produced spatial distribution map showed that 21.71% of the study area was non-saline, 29.78% was slightly saline, 31.40% was moderately saline, 15.25% was strongly saline and 1.44% was very strongly saline. The multivariate linear regression analysis provided more successful results in determining soil salinity. The results showed the importance of vegetation and salinity indices for modeling and mapping soil salinity, applying effective soil improvement methods and monitoring the change of soil salinity over time. The results obtained in this study are useful for monitoring and reclamation of soil salinity of agricultural lands in arid regions.
